The article "Predicament and Outlet: The Deep Fusion of Information Technology and Political Thought Teaching in Institution of Higher Learning under the Background of Fragmented Learning Environment" was retracted in 2023. Reasons: signs of a paper mill; suspected computer-generated content; unreliable results or conclusions; concerns about the data.

# Predicament and Outlet: The Deep Fusion of Information Technology and Political Thought Teaching in Institution of Higher Learning under the Background of Fragmented Learning Environment

**DOI:** 10.1155/2022/3177706

**Published:** 2022-09-08

**Authors:** Xueqiu Wen

**Affiliations:** Guangdong Polytechnic of Water Resources and Electric Engineering, School of Marxism, Guangzhou 510925, China

## Abstract

The ongoing integration of IT with various disciplines is a result of IT's constant penetration of the educational sector. This paper investigates how to further promote the deep integration of IT and political thought courses in institution of higher learning based on the fragmented learning background, starting from the current teaching situation of political thought courses in institution of higher learning, based on modern educational theory and supported by IT. Strengthening the relevance and affinity of political thought courses in institutions of higher learning and more effectively implementing the political thought instructional resource are examples of new approaches that can be explored to increase the effectiveness of political thought education and teaching. The integration model of political thought course instructional resources in higher education institutions is also constructed in this paper. According to the user's interest characteristics, the instructional resources are filtered, and the search service and recommendation service of political thought instructional resources are few but adequate. This model introduces personalized information service based on network into the instructional resource system, learning, and tracking users' personalized interests. The results of the experiments demonstrate that this algorithm has an accuracy of up to 95.03 percent. IT has a certain degree of applicability and dependability, and this study can offer valuable reference material for the deep integration of IT and political thought teaching in institutions of higher education against the backdrop of fragmented learning.

## 1. Introduction

Information technology (IT) has rapidly advanced, causing profound changes in people's lives, as well as altering their educational and social norms and fostering a more open society. Modern IT development is a requirement for modern education, and both modern IT theory and modern educational theory are essential components of modern teaching [1]. Contemporary educational practice has increasingly shown that modern IT and education and teaching of various disciplines are showing a trend of increasing integration. Political thought theory course is an important part of higher education system. The scientific nature of the theory of political thought courses in institution of higher learning is essentially reflected in the scientific nature of the guiding ideology [2]. By studying Marxist theoretical viewpoints, students can establish correct values, outlook on life, and world outlook. In the process of rapid development, IT has been continuously integrated into various fields of society, and the constant penetration of IT in the field of education has promoted the integration of IT and education and teaching. IT is gradually introduced into the political thought teaching in institution of higher learning. Network resources enrich the teaching content of political thought courses in institution of higher learning and are an important way to effectively achieve the instructional resource of political thought courses in institution of higher learning [3]. Political thought courses have been steadily enhancing the teaching materials and refining the curriculum design in higher education institutions for many years. As a result, a relatively logical, scientific, and stable curriculum system has developed. Currently, higher education institutions have dedicated a certain amount of manpower, material resources, and financial resources to building multimedia and network-based political thought courses. There is still a significant gap between utilizing IT fully in political thought education and teaching, though [4]. Many educators are starting to focus more on how to integrate contemporary IT with teaching and learning because of the powerful support it can give to educational reform. IT can be used to change educational practices, which will improve and strengthen the impact of education and teaching.

The article "Predicament and Outlet: The Deep Fusion of Information Technology and Political Thought Teaching in Institution of Higher Learning under the Background of Fragmented Learning Environment" was retracted in 2023. Reasons: signs of a paper mill; suspected computer-generated content; unreliable results or conclusions; concerns about the data.

At the moment, there is a dearth of in-depth research on the integration of IT and political thought education and teaching, particularly the theoretical research combined with specific implementation links. The emergence of new media and mobile communication technology has had a profound impact on people's communication styles, reading paradigms, and learning styles, as well as a shift from centralized to fragmented information dissemination in the new era of rapid economic and social development [5]. With the rise of the Internet, the term fragmentation has acquired new meaning. The effectiveness of political thought classes in institutions of higher learning is greatly impacted by knowledge fragmentation, information dissemination fragmentation, and lifestyle fragmentation, all of which interact and reinforce one another by primarily occupying students' time online and affecting their learning and thinking processes. In the new era of information exchange, fragmentation learning has emerged as a key component [6]. If the fragmented information obtained by college students cannot effectively supplement or correctly interpret the theoretical system of political thought courses in time, it will directly hinder students' scientific understanding of the theoretical system of political thought courses. Under the background of fragmented learning, we must adapt to the current situation of rapid development of network data [7]. Teachers of political thought courses should pool ideas. Use one's brains to change the teaching ideas, integrate the complicated network resources, and establish a resource bank suitable for political thought course teaching in institution of higher learning, in order to help teachers and students use resources in time and carry out more effective political thought teaching. In view of this, this paper discusses the deep integration of IT and political thought teaching in institution of higher learning under the background of fragmented learning. The innovations of the article are as follows:

① Innovation of research perspective. Information exchange in the new era now frequently includes fragmentation learning. This paper examines how to further encourage the thorough integration of IT and political thought teaching in institution of higher learning based on the fragmented learning background, starting from the current situation of political thought teaching in institution of higher learning, based on contemporary educational theory and supported by IT.
② Innovation of research methods. In the aspect of building user model, the system extracts the features of users' personalized resource access to form individual user model and cluster users with similar interests to form a group user model. Finally, the two user models are integrated to form an integrated user interest vector to build an integrated user model. At the same time, this model solves the problem of users' cold start by two-step training and realizes the personalized recommendation function of political thought education resources.

The article "Predicament and Outlet: The Deep Fusion of Information Technology and Political Thought Teaching in Institution of Higher Learning under the Background of Fragmented Learning Environment" was retracted in 2023. Reasons: signs of a paper mill; suspected computer-generated content; unreliable results or conclusions; concerns about the data.

## 2. Related Work

A key national educational development strategy and a current trend in education is the comprehensive integration of modern IT with contemporary teaching and learning. Promoting the thorough blending of IT and political thought education in institutions of higher learning has also developed into an important topic that many academics are now paying attention to. The understanding of how IT can be used to enhance learning and teaching has undergone a gradual and ongoing development process.

Zhu et al. believe that the integration of IT and contemporary education is a comprehensive and profound innovative change. It innovated the traditional education model and made profound changes in teaching methods, teaching tools, and teaching content [8]. Starting from the course nature of political thought courses in institution of higher learning, Song uses the dialectical relationship between form and content and purpose and means to analyze the possibility of deep integration of IT and political thought teaching in institution of higher learning [9]. Zhu pointed out that network resources in the context of the data age are a double-edged sword. While this brings help to teaching, it also increases risks, making teachers face the challenge of integrating network resources for political thought courses in institution of higher learning. Therefore, when developing and utilizing network resources, principles should be followed to avoid blindness [10]. Yu and Wang proposed that, in the face of the impact of fragmented learning on political thought courses, institution of higher learning needs to change their teaching thinking, face up to new methods of fragmented learning, innovate teaching methods, and give full play to the advantages of network platforms; focus on teaching links and achieve fragmented learning organic combination with systematic learning; improve the way of course assessment and enhance the comprehensive ability of college students; and improve the teaching effectiveness of political thought theory courses in institution of higher learning [11]. Su analyzes the realistic dilemma of fragmented learning of political thought courses in the new era, interprets its causes, and gives countermeasures. It is expected to provide useful management information for improving the teaching effect of political thought courses and the quality of personnel training [12]. Liang pointed out that the deep integration of IT and the teaching of political thought courses in institution of higher learning is not completely dominated by IT, nor is it to engage in formalism; instead, it is necessary to better play the educational value of IT and use IT means to enhance political thought courses. The affinity and pertinence of the course truly stimulate the enthusiasm of students to study political thought courses [13]. Du believes that, in the existing research, there are three main research methods for the deep integration of IT and education: regional construction, network learning, and classroom teaching [14]. Ma proposed increasing the attention to the fragmented information that students are most concerned about. Institution of higher learning should pay close attention to the fragmented information that students often receive and activate a dynamic supervision mechanism when necessary to properly supervise and influence [15]. Li and Zheng proposed that the countermeasures to enhance the effectiveness of political thought classrooms in institution of higher learning under the background of knowledge fragmentation mainly include leveraging on fragmentation and improving the quality of political thought classrooms, guiding fragmentation, gradually improving the depth of political thought classrooms, and transcending fragmentation, innovating, and expanding thinking political classroom space [16]. Xu and Tsai believe that the deep integration of IT and education faces three major problems. One is reflected in concepts and mechanisms; another is teachers and students; and the third is networks and resources [17].

The article "Predicament and Outlet: The Deep Fusion of Information Technology and Political Thought Teaching in Institution of Higher Learning under the Background of Fragmented Learning Environment" was retracted in 2023. Reasons: signs of a paper mill; suspected computer-generated content; unreliable results or conclusions; concerns about the data.

In general, there is not enough current research on the thorough blending of IT and political thought education. Based on this, the paper discusses the intricate integration of IT and political thought instruction in higher education institutions against the backdrop of fragmented learning. In this paper, against the backdrop of knowledge fragmentation, thoroughly integrating IT with political thought teaching in higher education institutions is proposed in order to increase the effectiveness of political thought classrooms in institutions of higher learning and provide references for doing so. In addition, this paper builds the instructional resource model for a higher education institution's political thought course. The study demonstrates that this model is capable of realizing the personalized recommendation function of political thought education resources and effectively resolving the issue of users' cold starts.

## 3. Methodology

### 3.1. Deep Integration with Political Thought Teaching in IT Universities

Under the direction of the fundamental concepts and procedures of information science, IT is a technology that enhances human information function. IT, in general, refers to a collection of technologies that use computers and contemporary communication as their primary tools for acquiring, processing, transmitting, and utilizing information. It consists of four fundamental technologies: control technology, computer technology [18], communication technology, and sensing technology. The constant penetration of IT in the field of education makes IT continuously integrate with various disciplines. The advent of modern IT inevitably has a great influence on the traditional political thought education in institution of higher learning. IT is an activity to educate human beings to use IT to achieve educational purposes [19]. Education cannot be separated from IT, and IT itself is also an important part of education, and the education and teaching of political thought course are no exception. Political thought courses in institution of higher learning are responsible for studying, researching, and imparting Marxist theoretical knowledge and cultivating students' socialist core values and ideals and beliefs. The development of IT and its application in education are the result of choice and adaptation. With the support of IT, young students can get in touch with more new things with the help of new media. This can not only broaden their horizons and make them receive more valuable information but also promote personal growth and guide them to form a correct understanding of political thought education. The learning environment under IT is no longer limited by the traditional physical space but is integrated with the traditional learning environment. The learning environment under IT has the advantages of sharing, interaction, advancement, and renewability. As the forefront of training all kinds of national talents, institution of higher learning must always keep pace with the times and do a good job of using advanced technology to guide teaching. Information-based teaching means should exert not only its explicit instrumental value but also its implicit educational value and unify its instrumental and educational values. With the deepening of the integration of IT and political thought education and teaching, some potential problems and practical puzzles are gradually revealed [20]. For example, IT is only used as a tool for knowledge transmission, while its cognitive tools and intellectual tools are ignored. To some extent, this affects the effective application of IT in political thought teaching in institution of higher learning. The function and application of IT in political thought teaching are shown in Figure 1.

The article "Predicament and Outlet: The Deep Fusion of Information Technology and Political Thought Teaching in Institution of Higher Learning under the Background of Fragmented Learning Environment" was retracted in 2023. Reasons: signs of a paper mill; suspected computer-generated content; unreliable results or conclusions; concerns about the data.

As far as the political thought course teaching itself is concerned, there are the following structural problems: ① The level of teachers is uneven, and teachers lack incentive mechanism. ② The implementation of large class teaching makes students' learning motivation insufficient. ③ There is less interaction between teachers and students, and there is a certain distance between teaching materials and reality. At present, the role of IT in education and teaching is paid more and more attention. The majority of political thought teachers have realized the importance of effective application of IT in political thought education and teaching. In the construction of multimedia teaching and network teaching of political thought course, institutions of higher learning all over the country have invested a certain amount of manpower, material resources, and financial resources and achieved certain results. Political thought courses must be subject to an efficient supervision mechanism in order to have the desired effect. The teaching content of political thought courses can be strengthened even more by adapting the information-based teaching format to it in higher education institutions. The information-based teaching method can therefore be further enhanced by the teaching of this course material [21]. Additionally, the teaching of this course can be promoted more successfully through the use of IT virtual space, which can investigate a wider field and broaden the position on the course's original basis. A wealth of global information and significant interactive resources have been made possible by the quick development of IT. Many different pieces of information are sent out on a daily basis from various network platforms, and the network resources are updated in real time with high speed, short cycle, and high mobility. Through various network channels, people can disseminate the most recent information, and the transmission rate is very quick. For college students, it is extremely important to broaden their knowledge bases, increase their social networks, and improve their academic lives. Additionally, it improves the depth, complexity, and efficacy of political thought education in institutions of higher learning. Under the IT environment, the cooperative teaching mode of political thought courses in institution of higher learning is helpful to cultivate students' subjective consciousness, self-comprehension, self-evaluation, and self-regulation ability and habits, so that students can learn how to learn through independent inquiry activities, and students at different levels can actually improve their basic academic ability, developmental academic ability, and innovative academic ability.

At present, fragmented information is widely spread, and various ideological cultures collide and blend, which brings severe challenges to the political nature of the theory of political thought courses. For college students, under the influence of this fragmentation, the fragmentation of their knowledge is more closely related to it. Objectively speaking, fragmentation is a double-edged sword. Fragmentation learning is to break down the whole content into easy-to-understand parts, and the information, knowledge, and other contents are fragmented. Although it adapts to the purpose that college students can use their spare time to learn flexibly according to their own learning needs and learning progress anytime and anywhere, it makes knowledge become illogical and organized, and information becomes scattered and disorderly. The fragmentation of knowledge brings about the incompleteness of knowledge system. Therefore, political thought educators should explore ways to go beyond the fragmentation and strive to expand the classroom space of political thought education. In the era of information fragmentation, political thought teachers and educational administrators should learn from the rational and scientific nutrients of other discourse systems with a more open and inclusive mind. In this process, we will make full use of high-tech such as big data and cloud computing to comprehensively improve the effectiveness of fragmented learning of political thought courses. Under the background of fragmented learning, classroom teaching is no longer the only way to impart knowledge. The ways for students to obtain information are increasingly extensive, and the space for receiving information is constantly expanding. At ordinary times, political thought teachers should go deep into the students after class to know the fragmented information about political phenomena and social hot issues that students are most concerned about and then select the appropriate fragmented information about politics as a topic in combination with students' opinions. Through discussion and communication with others, students can naturally sum up theoretical conclusions. The systematic study of political thought course in institution of higher learning is to explain the content in a fixed time and place, emphasizing the integrity and continuity of knowledge, so that college students can establish a systematic knowledge framework. Faced with the situation of fragmented learning, the educators of political thought courses in institution of higher learning can promote the deep integration of IT and political thought courses if they can use modern IT correctly, appropriately, reasonably, and timely. This is bound to greatly improve the effectiveness of political thought education and teaching, thus improving the quality and level of political thought education and teaching.

The article "Predicament and Outlet: The Deep Fusion of Information Technology and Political Thought Teaching in Institution of Higher Learning under the Background of Fragmented Learning Environment" was retracted in 2023. Reasons: signs of a paper mill; suspected computer-generated content; unreliable results or conclusions; concerns about the data.

### 3.2. Construction of Instructional Resources of Political Thought Courses in Institution of Higher Learning

The varieties of network information content are numerous, varied, and colourful. However, the diversification of network resources brings about the mingling of unfavourable images, which affects students' ideological and moral consciousness and hinders their ability to develop good values. Therefore, it is important to incorporate a variety of instructional resources into online education resources that also contain the right principles for building social and spiritual civilizations and to help students develop the right attitudes and values. The improvement of the network of instructional resources for political thought theory courses in institutions of higher learning, as well as the conduct of research on solutions, is of great theoretical significance and practical value. A service that caters to users' individual needs for instructional resources based on their usage patterns and personality traits is known as a personalised instructional resource service. We must take into account the multilevel, diversified, open, and dynamic updating timeliness of the resource library construction when building the resource library in order to ensure that various learners can access the resources they require. This is because learners have individual differences in learning starting points, learning styles, learning desires, learning pace, and so forth. The construction of IT teaching environment is shown in Figure 2.

Individualized characteristics of users refer to the combination of characteristic information of their demand for instructional resources determined by individual characteristics, that is, a series of useful information generated by the decisive relationship of specific users' demand for instructional resources. Personalized recommendation recommends information that users are potentially interested in, thus improving the efficiency of information acquisition. In addition, personalized recommendation can also guide users' information needs, fully tap users' potential interests, and help them discover new interests. Users' feedback on recommendation information can dynamically update the interest model of the subject, so as to provide the subject with various information products that can best meet its needs. Using user's personality information has the three following functions: ① User's personality information is used to standardize and modify user's query request. ② It is used to guide the acquisition of information by processing query requests and user personality information. ③ The information of user's personality is used to process the query results. Users can actively provide personal interests to the recommendation system, including explicit information and implicit information of users. The recommendation system automatically matches the user's personal preferences into the preference information base, and the recommendation engine automatically provides personalized recommendations to users by querying the user's access mode information in the preference information base and related databases in the resource database and using the corresponding personalized recommendation strategy. The algorithm of similarity calculation is mainly used to calculate the similarity between users or projects. Taking the calculation of item similarity as an example, its generality lies in that the common scoring users are selected for the two items *i* and *j* from the scoring or other user preference matrixes, and then the similarity *S*_*i*,*j*_ is calculated for the two common scoring vectors. Cosine similarity specifically refers to the cosine angle between two different vectors. Let the vectors $\overset{⟶}{i}$ and $\overset{⟶}{j}$ be expressed as *n*-dimensional vectors; namely,

(1) $$\begin{array}{c} i=\left\{i_{1},i_{2},i_{3},\ldots ,i_{n}\right\},\\ j=\left\{j_{1},j_{2},j_{3},\ldots ,j_{n}\right\}. \end{array}$$

The cosine similarity calculation method is as follows:

(2) $$\begin{array}{c} \text{Sim}\left(i,j\right)=\text{cos}\left(\overset{⟶}{i},\overset{⟶}{j}\right)\frac{\overset{⟶}{i}\cdot \overset{⟶}{j}}{\left|\overset{⟶}{i}\right|\cdot \left|\overset{⟶}{j}\right|}. \end{array}$$

Pearson correlation coefficient is also called correlation similarity. Suppose that we use *U*={*u*_1_, *u*_2_, *u*_3_,…, *u*_*n*_} to represent the set of users and *I*={*i*_1_, *i*_2_, *i*_3_,…, *i*_*n*_} to represent the set of items. The specific calculation method for calculating item similarity is as follows:

(3) $$\begin{array}{c} \text{Sim}\left(i,j\right)=\frac{\sum_{u\in U_{ij}}\left(r_{ui}-\bar{r_{i}}\right)\left(r_{uj}-\bar{r_{j}}\right)}{\sqrt{\sum_{u\in U_{uj}}{\left(r_{ui}-\bar{r_{i}}\right)}^{2}}\sqrt{\sum_{u\in U_{uj}}{\left(r_{uj}-\bar{r_{j}}\right)}^{2}}}. \end{array}$$

At the same time, the similarity between different users can also be calculated. The calculation method is as follows:

(4) $$\begin{array}{c} \text{Sim}\left(u,v\right)=\frac{\sum_{i\in I_{uv}}\left(r_{ui}-\bar{r_{u}}\right)\left(r_{vi}-\bar{r_{v}}\right)}{\sqrt{\sum_{i\in I_{uv}}{\left(r_{ui}-\bar{r_{u}}\right)}^{2}}\sqrt{\sum_{i\in I_{uv}}{\left(r_{vi}-\bar{r_{v}}\right)}^{2}}}. \end{array}$$

Users have various interests, and they can choose appropriate keywords to express their interests according to the instructional resources they have browsed. Then the instructional resources containing these words are regarded as instructional resources that satisfy users' interests, that is, relevant instructional resources. The establishment of user's interest model is a dynamic and constantly adjusting process, which is always in progress. During the interaction with users, the recommendation system will actively record users' historical interest information, model users' information needs, form a knowledge model about users' interests and preferences, and realize the final information recommendation service according to this model. In mathematics, linear correlation coefficient refers to two variables with linear correlation. When one variable gets bigger, the other variable will get bigger. On the other hand, if one variable decreases, the other will also decrease. The accuracy will decrease if the similarity is determined using the user scoring matrix because it will have a significant negative impact on performance. It is challenging to precisely calculate the similarity of two vectors when the data is sparse because the similarity calculation is primarily based on finding similar objects or users. The empty spaces in the user's scoring matrix are typically filled with data to address the issue of sparse data. After using the vector space model to represent the characteristics of the document, the user's interest can be regarded as a document, which can also be expressed as a vector *U*. The similarity between the document and the user's interest can be represented by the cosine similarity Sim(*V*, *U*) between the document vector *V* and the user's interest vector *U*. The average weighted score of user *i* is calculated as shown in the following formula:

(5) $$\begin{array}{c} r_{u}=\bar{r_{u}}+\frac{\sqrt{\sum_{k=1}^{k}{\left(r_{k,i}-\bar{r_{i}}\right)}^{2}}}{K}. \end{array}$$

In the above formula, *K* is the total number of ratings of item *i* by user; *r*_*k*,*i*_ is the rating value of the unrated item *i* by user *k*. The average weighted score of item *i* is calculated as shown in the following formula:

(6) $$\begin{array}{c} r_{i}=\bar{r_{i}}+\frac{\sqrt{\sum_{q=1}^{Q}{\left(r_{u,q}-\bar{r_{i}}\right)}^{2}}}{Q}. \end{array}$$

In the above formula, *Q* is the total number of ratings of user *u* to the item space; *r*_*u*,*q*_ is the rating value of *k* to user *u* to *q*. Then, the weighted score is integrated to get the following formula:

(7) $$\begin{array}{c} r_{u,i}=\alpha r_{u}+\beta r_{i}\alpha +\beta =1. \end{array}$$

In this way, the integrated weighted score of the unscored items is obtained and the corresponding items are filled. Any item in the matrix has a score for items *i* and *j*, and the contribution judgment parameters *α* and *β* are introduced. The integrated weighted score is determined by the user's subjective score and the item's objective score. The score factor is composed of two parts, and the contribution of the two in the whole formula is different, because adding the judgment parameter makes the recommendation result more accurate.

The article "Predicament and Outlet: The Deep Fusion of Information Technology and Political Thought Teaching in Institution of Higher Learning under the Background of Fragmented Learning Environment" was retracted in 2023. Reasons: signs of a paper mill; suspected computer-generated content; unreliable results or conclusions; concerns about the data.

Students and teachers make up the majority of users of the instructional resource sharing module. The resources are available for browsing, searching by category, searching by keyword, uploading, and downloading, as well as being rated and commented on by students and teachers, allowing them to determine the resources' value in a fair and reasonable manner. Teachers can manage all uploaded resources, edit them, and delete them. Teachers can review and edit the resources that students upload, publish them to the resource database, and ensure that they are of a high calibre. The application of the recommendation algorithm module is the recommendation function. The same recommendation algorithm can be used for multiple recommendation functions and the same recommendation function can be used for multiple recommendation algorithms. Two personalized recommendation functions are realized in this paper by the personalized recommendation module: automatic recommendation of new instructional resources and user request recommendation. Among them, the automatic recommendation of new instructional resources is essentially a kind of personalized retrieval, that is, the retrieval of new instructional resources collected by the system during the period when users have not used the system. The user's request for recommendation is realized by calling the instructional resource management module and the instructional resource filtering module. In a single machine environment, it takes a long time to calculate recommendations from large amounts of data, and stack overflow can happen. However, the enhanced MapReduce-based parallel recommendation algorithm distributes a sizable amount of computation across numerous Map nodes to make up for Hadoop's transmission consumption after changing and rearranging the data structure. The parallelized algorithm performs better overall than running the algorithm on a single machine, which is obviously better. As a result, the system supports simultaneous access from a large number of users, can handle high concurrent requests, and has good stability. In order to provide users with a positive user experience, it is also necessary to have a friendly, succinct, and beautiful interface, strong robustness, simple and understandable software, easy maintenance and expansion, simple user operation, and strong versatility.

## 4. Result Analysis and Discussion

After the realization of the instructional resource model, the next step is to design an evaluation experiment for this model, so as to quantitatively obtain all the indicators of the model. In this way, we can have a deeper understanding of the advantages and disadvantages of the model and at the same time provide a reference for the optimization of model parameters and the further optimization of the model. There are naturally differences in the effect of the system to achieve the filtering goal, and a set of standards are needed to evaluate its effect. At present, there is no unified or reasonable standard. First of all, the filtering system not only faces the information content but also contains many social factors. Secondly, users' interests are diverse, and their connotations are not uniform and fixed. Different users have different understandings of the same word, which will lead to different evaluations of the filtering results.

The article "Predicament and Outlet: The Deep Fusion of Information Technology and Political Thought Teaching in Institution of Higher Learning under the Background of Fragmented Learning Environment" was retracted in 2023. Reasons: signs of a paper mill; suspected computer-generated content; unreliable results or conclusions; concerns about the data.

MAE (mean absolute error) is measured by calculating the error between the predicted user rating and the actual user rating. Mainly combined with cross-validation, the formula is as follows:

(8) $$\begin{array}{c} \text{MAE}=\frac{\sum_{g^{\text{test}}\subset G^{\text{test}}}\left|g^{\text{test}}\left(\text{prediction}\right)-g^{\text{test}}\left(\text{authentic}\right)\right|}{\left|G^{\text{test}}\right|}. \end{array}$$

In the above formula, *g*^test^(authentic) is the real score, *g*^test^(prediction) is the predicted score, and *G*^test^ is the entire set of user scores to be predicted. A single value indicator called average accuracy shows how well the system performs across all pertinent documents. The higher the average accuracy, the more relevant documents the system is able to retrieve. The equation reads as follows:

(9) $$\begin{array}{c} \text{MAP}=\frac{1}{\left|U\right|}\sum_{i=1}^{\left|U\right|}\frac{1}{\left|R_{i}\right|}\sum_{j=1}^{\left|R_{i}\right|}\frac{j}{r_{ij}}. \end{array}$$

In the above formula, *U* is the set of test users; |*U*| is the number of test user sets. The following experiment shows the MAE of different algorithms as shown in Figure 3. The average accuracy of different algorithms is shown in Figure 4.

If the system gathers new instructional resources while the user is not using the system and if the user requests a recommendation after logging in, the purpose of the instructional resource recommendation module is to recommend new instructional resources in the form of newly uploaded instructional resources. The performance of the system may be impacted if the personalized recommendation module of learning resources directly adopts the investigated algorithm due to excessive calculation. Consequently, it is important to take algorithmic performance optimization into account when putting the recommendation algorithm into practice. The performance of the recommended algorithm before and after optimization is shown in Figure 5.

Under the condition that the Top-N value is 25, the performance indexes of the algorithms before and after optimization are compared and analyzed. Performance evaluation indexes mainly include accuracy, recall, and coverage.  Table 1 shows the experiment of each index.

The article "Predicament and Outlet: The Deep Fusion of Information Technology and Political Thought Teaching in Institution of Higher Learning under the Background of Fragmented Learning Environment" was retracted in 2023. Reasons: signs of a paper mill; suspected computer-generated content; unreliable results or conclusions; concerns about the data.

From the comparison of results, it can be seen that the performance of the improved algorithm is slightly higher than that of the basic collaborative filtering algorithm, which further proves the value of the experiment.

The recall rate is the ratio of the total number of objects preferred by users in the recommendation result set to the number of all objects preferred by users in the system. Let *R*(*u*) represent the number of object resources preferred by the user in the recommendation result set; and let *T*(*u*) be the number of all object resources that the user prefers in the system. Then the recall rate is

(10) $$\begin{array}{c} \text{Recall}=\frac{R\left(u\right)}{T\left(u\right)}\times 100\%. \end{array}$$

In the above formula, *T*(*u*) is the number of all objects in the recommended result set. The comparison of recall rates of different algorithms is shown in Figure 6.

This system uses a vector space model to represent user templates and documents, and its matching technology uses this model to determine how far apart two documents are from one another. In order to receive feedback, users must express a clear binary judgment about the provided instructional resources, that is, satisfied or dissatisfied. The outcome is then used to increase the proportion of feature items, which affects the similarity. In order to prevent operations from being left unfinished and to guarantee the consistency and integrity of the data in the database, operations like inserting, updating, and deleting require transaction management. Evaluation algorithm is crucial because it serves as a benchmark for gauging the effectiveness of recommendations made by recommendation systems. Therefore, in order to thoroughly evaluate the recommendation effect of a recommendation system, the selection of evaluation algorithms as well as the characteristics of various evaluation algorithms must be taken into consideration. In this paper, experiments are conducted again, and the accuracy of resource recommendation of different algorithms is shown in Figure 7.

In addition, in order to record and track users' personalized information about instructional resources in time, this paper designs a database of users' personalized features, which is used to store the keywords of instructional resources that users are most interested in and their access time.  Table 2 shows the user rating of the system.

It can be seen that, compared with the original system, this system has more friendly interface, concise and beautiful appearance, simple software, simple user operation, and strong versatility, which can give users a good user experience.

The article "Predicament and Outlet: The Deep Fusion of Information Technology and Political Thought Teaching in Institution of Higher Learning under the Background of Fragmented Learning Environment" was retracted in 2023. Reasons: signs of a paper mill; suspected computer-generated content; unreliable results or conclusions; concerns about the data.

The teaching of political ideology is deeply entwined with IT in IT universities, which not only pay attention to making the most of educational resources and environments but also pay attention to the benefits and drawbacks of IT teaching and learning, as well as how to compensate for the shortcomings. Put your attention on finding solutions to issues with open resource sharing, teacher-student cooperation and interaction, environment creation and renewal, innovative teaching model development, and other issues. The experiments in this chapter demonstrate that the algorithm's accuracy can reach 95.03 percent. It is reliable and practical in some ways. The system can efficiently provide a recommendation engine, analyze user behaviour and educational resources in a timely manner, build corresponding models, and address cold start and data sparsity issues. The system also allows for dynamic adjustments to database size or data volume, such as periodic resource maintenance by administrators, the ingesting of high-quality resources, and the deletion of low-quality resources. The system is adaptable to various operating environments and customer requirements due to the layered architecture design.

## 5. Conclusions

Today's world is undergoing a major trend toward digitization, which is a powerful force behind many of the economic and social changes that are occurring. The level of information technology in a country is now a crucial indicator of its overall strength and competitiveness. Information education should be a priority in the 21st century's education. Modern IT development is a requirement for modern education, and modern IT theory itself, along with modern educational theory, directly becomes an integral part of modern teaching. In other words, it would be extremely difficult to accomplish the goals and objectives of education and teaching without contemporary IT theories and tools. However, the advent of the fragmentation era has had a significant impact on political thought education. The fragmentation of knowledge, the fragmentation of lifestyle, and the fragmentation of information dissemination all work in concert to influence the political thought education system in higher education institutions. Based on this, the paper discusses the intricate integration of IT and political thought instruction in higher education institutions against the backdrop of fragmented learning. Additionally, it is advised that political thought teachers in institutions of higher education should judiciously implement the fragmented learning approach and actively research new methods of political thought teaching; strengthen college students' understanding of the value of book knowledge; strengthen the overall impact of political thought education; and strengthen the development of political thought teachers in order to increase the allure of political thought. Additionally, this paper develops a model for integrating instructional materials for political thought courses in institutions of higher education. By using a two-step training process, this model addresses the issue of users' cold starts. The results of the experiments demonstrate that this algorithm has a 95.03 percent accuracy rate. It has a certain degree of viability and dependability. The personalized recommendation of political thought instruction resources offered by this model is a good one. The research has some practical implications as a result. The model's performance will be continually enhanced and discussed in more detail.

The article "Predicament and Outlet: The Deep Fusion of Information Technology and Political Thought Teaching in Institution of Higher Learning under the Background of Fragmented Learning Environment" was retracted in 2023. Reasons: signs of a paper mill; suspected computer-generated content; unreliable results or conclusions; concerns about the data.

## Figures and Tables

**Figure 1:** The function and application of IT in political thought teaching.

**Figure 2:** Schematic diagram of instructional resources and environment construction under IT.

**Figure 3:** MAE situation of different algorithms.

**Figure 4:** Average accuracy of different algorithms.

**Figure 5:** Comparison of the performance of recommended algorithms before and after optimization.

**Figure 6:** Comparison of recall rates of different algorithms.

**Figure 7:** Comparison of resource recommendation accuracy of different algorithms.

**Table 1:** Experimental results of each index before and after optimization.

Algorithm	Accuracy rate (%)	Recall rate (%)	Coverage rate (%)
Basic collaborative filtering algorithm	85.64	86.31	79.63
Algorithm in this paper	93.27	95.27	89.76

**Table 2:** User rating of the system.

Evaluating indicator	Student user (%)	Teacher user (%)
Aesthetics of interface	93.94	92.17
Ease of operation	92.56	95.97
Search resource accuracy	92.11	90.38
Recommended resource accuracy	93.24	92.68
Goodwill	90.23	93.16

## Data Availability

The data used to support the findings of this study can be obtained from the author upon request.
